# Combining cell therapy with human autologous Schwann cell and bone marrow-derived mesenchymal stem cell in patients with subacute complete spinal cord injury: safety considerations and possible outcomes

**DOI:** 10.1186/s13287-021-02515-2

**Published:** 2021-08-09

**Authors:** Saeed Oraee-Yazdani, Mohammadhosein Akhlaghpasand, Maryam Golmohammadi, Maryam Hafizi, Mina Soufi Zomorrod, Nima Mohseni Kabir, Maryam Oraee-Yazdani, Farzad Ashrafi, Alireza Zali, Masoud Soleimani

**Affiliations:** 1 Functional Neurosurgery Research Center, Shohada Tajrish Comprehensive Neurosurgical Center of Excellence, Shahid Beheshti University of Medical Sciences, Tehran, 1988873554 Iran; 2 Stem Cell Technology Research Centre, Tehran, Iran; 3 Department of Research and Development, Sodour Ahrar Shargh Company, Tehran, Iran; 4 Applied cell Sciences Department, Faculty of Medical Sciences, Tarbiat Modares University, Tehran, Iran; 5 Department of Neurosurgery, Imam Hossein Hospital, Shahid Beheshti University of Medical Sciences, Tehran, Iran; 6 Department of Hematology, Tarbiat Modares University, Tehran, Iran

**Keywords:** Subacute complete spinal cord injury, Combination cell therapy, Schwann cells, Bone-marrow-derived mesenchymal stem cell

## Abstract

**Background:**

Cellular transplantations have promising effects on treating spinal cord injury (SCI) patients. Mesenchymal stem cells (MSCs) and Schwann cells (SCs), which have safety alongside their complementary characteristics, are suggested to be the two of the best candidates in SCI treatment. In this study, we assessed the safety and possible outcomes of intrathecal co-transplantation of autologous bone marrow MSC and SC in patients with subacute traumatic complete SCI.

**Methods:**

Eleven patients with complete SCI (American Spinal Injury Association Impairment Scale (AIS); grade A) were enrolled in this study during the subacute period of injury. The patients received an intrathecal autologous combination of MSC and SC and were followed up for 12 months. We assessed the neurological changes by the American Spinal Injury Association’s (ASIA) sensory-motor scale, functional recovery by spinal cord independence measure (SCIM-III), and subjective changes along with adverse events (AE) with our checklist. Furthermore, electromyography (EMG), nerve conduction velocity (NCV), magnetic resonance imaging (MRI), and urodynamic study (UDS) were conducted for all the patients at the baseline, 6 months, and 1 year after the intervention.

**Results:**

Light touch AIS score alterations were approximately the same as the pinprick changes (11.6 ± 13.1 and 12 ± 13, respectively) in 50% of the cervical and 63% of the lumbar-thoracic patients, and both were more than the motor score alterations (9.5 ± 3.3 in 75% of the cervical and 14% of the lumbar-thoracic patients). SCIM III total scores (21.2 ± 13.3) and all its sub-scores (“respiration and sphincter management” (15 ± 9.9), “mobility” (9.5 ± 13.3), and “self-care” (6 ± 1.4)) had statistically significant changes after cell injection. Our findings support that the most remarkable positive, subjective improvements were in trunk movement, equilibrium in standing/sitting position, the sensation of the bladder and rectal filling, and the ability of voluntary voiding. Our safety evaluation revealed no systemic complications, and radiological images showed no neoplastic overgrowth, syringomyelia, or pseudo-meningocele.

**Conclusion:**

The present study showed that autologous SC and bone marrow-derived MSC transplantation at the subacute stage of SCI could reveal statistically significant improvement in sensory and neurological functions among the patients. It appears that using this combination of cells is safe and effective for clinical application to spinal cord regeneration during the subacute period.

## Introduction

Spinal cord injury (SCI) is a devastating condition that leads to physical, social, and vocational impairment due to the irreversible loss of neural function below the injury site [1]. Based on *Lancet Neurology*, the global burden of diseases (GBD), injuries, and risk factors between 1990 and 2016, the age-standardized incidence of SCI was 13 per 100,000. Furthermore, with global population growth, the absolute number of people living with the effects of SCI is expected to increase [2]. Most of the SCI patients suffer from a profound disability and its related complications, which impact the quality of life [3]. Therefore, functional improvement after SCI remains an important issue in recent decades. Regarding the lack of capacity for central nervous system regeneration, there is no definitive cure for these disorders. Advanced therapies like cell transplantation could be a promising option for treating SCI patients [4].

Numerous studies on animal models of SCI and human patients have demonstrated that cellular transplantations for SCI treatment might provide a source of neural cells and have neuroprotective and immunomodulatory effects after injury [5, 6]. Various cell types can be used due to their capacity for self-renewal and differentiation ability, but among them, mesenchymal stem cells (MSCs) and Schwann cells (SCs) have better safety alongside their complementary characteristics, so these cells are suggested to be one of the best candidates for transplantation in SCI subjects [7, 8].

Bone marrow MSC as a multipotent stromal cell has a potential effect to differentiate into osteoblast, adipocytes, chondrocytes, mature neurons, and glial cells [9]. Many studies have shown that MSCs could be considered for the SCI treatment. Zhu et al. conducted a phase I–II clinical trial on 28 chronic complete SCI patients to assess the safety and efficacy of umbilical cord blood mononuclear cell transplant. They concluded that transplantation could be safe and would lead to locomotor, bowel, and bladder recovery [10]. Also, Ghobrial and colleagues enrolled 12 patients with traumatic SCI in a phase II safety and efficacy study of intramedullary injections of human neural stem cells. They presented five total patients with 12 months of follow-up and observed that transplantation can be safely performed with improvement in overall mean functional outcomes measures [11]. Moreover, MSCs can produce various types of growth factors and neuroprotective cytokines which enable them to improve or restore damaged spinal cord function [12–14]. Despite the beneficial effects of MSC transplantation, according to the previous findings, their remyelinating ability is inadequate in SCI patients. The importance of remyelination in spinal cord repair after injury suggests that stem cells could be combined with remyelinating cells to improve the effectiveness of transplantation [15]. SCs which are normally located in the peripheral nerves could migrate and colonize in lesion sites to myelinate injured axons and are one of the suitable choices for transplantation in combination with MSCs [16–18].

Successful functional recovery in the patients suffering from SCI will most likely rely on effective treatment in the period corresponding with the natural history of neuro recovery. The clinical trials have been conducted to assess the possible outcome of combinational cell therapy for treating patients with chronic SCI. Like our previous study, they have indicated an insufficient recovery in patients with chronic disease [8, 15]. So, in this study, we aimed to assess the safety and possible outcomes of co-transplantation of autologous bone-marrow MSC and SC in the patients with subacute traumatic complete SCI (within 12 months post-injury) [19].

## Patients and methods

### Study design and selection criteria

This study was designed on the basis of the Declaration of Helsinki and approved by Ethics in Medical Research Committee, Shahid Beheshti University of Medical Sciences (code of ethics: 106, approved in October 2011). All the interventions were performed after obtaining informed consent from patients.

Our inclusion criteria for the study were as follows: (1) complete SCI (ASI A); (2) ≥ 3 and ≤ 12 months post-injury; (3) no improvement in sensory and motor scale after 3 months despite regular rehabilitation program; (4) absence of brain disease or psychological disorders; (5) no stenosis, tethering, syringomyelia, or compression in the magnetic resonance images (MRI) of the spinal cord taken at the beginning of the study; (6) absence of joint stiffness or pain, rashes, or any manifestation of rheumatologic disorders; and (7) aged between 18 and 60 years old.

Study exclusion criteria were (1) presence of any movement disorder not related to SCI; (2) a major complication such as urinary tract infection with sepsis, pneumonia, venous thromboembolism (deep vein thrombosis and pulmonary embolism), etc.; (3) fracture of upper or lower limbs leading to deformity and ankylosis; and (4) abnormal findings on baseline complete blood count.

Patients were selected from among those with spinal cord injury who referred to the neurosurgery clinic of Shohada Tajrish Hospital. Eleven patients (9 men and 2 women) with a mean age of 29.09 ± 9.41 years old met our inclusion and exclusion criteria and successfully enrolled in this study. Four cases of the patients had cervical and seven had thoracic lesions due to road traffic accidents and falls from the height (Table 1).

**Table 1:** Demographic, clinical features, motor, and sensory level changes of the patients

Patient number	Sex	Age (years)	Cause of injury	LOI	Interval between injection and trauma (months)	Motor level pre-treatment	Motor level 6 months after treatment	Motor level 12 months after treatment	Sensory level pre-treatment	Sensory level 6 months after treatment	Sensory level 12 months after treatment
1	Male	18	Accident	C4	3	C7	C7	C8	T4	T4	T4
2	Female	42	Accident	T3	7	T1	T1	T1	T3	T4	T4
3	Female	38	Accident	T10	3.5	L1	L1	L1	L1	L1	L1
4	Male	27	Accident	C5	5	C6	C7	C7	C5	C5	C5
5	Male	21	Accident	T12	9	T1	L3	L3	L5	L5	L5
6	Male	30	Accident	T6	5.5	T1	T1	T1	T8	T10	T10
7	Male	17	Falling	T5	3	T1	T1	T1	T5	T9	T9
8	Male	30	Accident	C5	4	C7	C7	C7	T2	T3	T3
9	Male	19	Accident	T2	7	T1	T1	-	T3	T3	T12
10	Male	40	Accident	T11	3	T1	T1	-	T12	T12	-
11	Male	38	Accident	C5	8	C7	C8	C8	C4	C4	C4

*LOI* level of injury

### Cell isolation and transplantation

All tests, including cell isolation and culture, were performed in Gandi Hospital’s cell therapy laboratory following Good Manufacturing Practice (GMP). Following the daycare procedure, the patients hospitalized, SCs, and MSCs were extracted from the patients in the operating room under sterile conditions, and they were discharged immediately after the procedure.

To collect SCs, as we previously reported [15], the sural nerve of the patient posterior to lateral malleolus was cut and sliced into 1- to 2-mm pieces, then was incubated with collagenase (1.4 U ml^−1^; Sigma, St. Louis, MO, USA) and Dispase (2.4 U ml^−1^; Sigma, USA). After washing the collagenase two times with DMEM/F12 and mesh filtering, the cells were treated with DMEM/F12, not including fetal bovine serum (FBS, Gibco, USA) for 5 days (37 °C, 5% CO_2_). After the fasting period, we gradually increased the concentration of FBS in culture progressively up to 10% during 1 week. The characterization of the isolated cells was approved by S-100 immunocytological staining, as described in our previous study [15].

To isolate bone marrow MSC, bone marrow blood (100–150 ml) was aspirated from the iliac bone. After the samples underwent a density gradient by Ficoll (1.077 g/l, Sigma, USA) at the ratio of 1:3, the mononuclear cell layer was recovered from the gradient interface after bone marrow blood was centrifuged (400*g* for 40 min). To separate the platelets and mononuclear cells, the cells were centrifuged three times with less gradient and time. To confirm that isolated cells were MSCs, we assessed the differentiation ability of these isolated cells to adipogenic and osteogenic cells. In addition, we assessed the cell surface markers (CD73, CD105, CD45, and CD34) through flow cytometry analysis to ensure the characteristic of the isolated cells which should be positive for CD73, CD90, and CD105 and negative for CD45.

MSCs and SCs were cultured and prepared separately then mixed before transplanting which was composed of MSCs at the final concentration of 5 × 10^7^ cells per ml and SCs at the final concentration of 5 × 10^7^ cells per ml. The cells were resuspended in 1 ml saline, and a total volume of 1 ml was injected into the SCI patient.

According to previous studies [12, 20, 21], transplantation was performed 3 weeks after cell harvesting, because 3 weeks is enough time to cultivate this number of cells. In this way, the cells were stored and cultured in the laboratory environment in the shortest possible time, and the cells have the highest quality at the time of transplantation. A physician transplanted the mixture of MSCs and SCs into the L4/L5 level in the operation room through lumbar puncture using spinal needle 24 G. We assured the entrance to the subarachnoid space by the existing CSF from the spinal needle. The mixture of cells (6 ml) was slowly injected. We kept the needle in place for 1 min to avoid leakage. The patients were discharged 1 h after the procedure.

### Quality control of MSCs

We use clinical-grade material from reputable companies such as Gibco. All cell operations were performed in a sterile environment to prevent possible contamination. GMP clean rooms for cells were designed to ensure the quality, safety, and efficacy of those biological treatments, which makes it extremely important to have a good monitoring system.

The existence of mycoplasma infection was investigated before and after antibiotic treatment using the PCR-based method. A universal generic-specific primer capable of detecting all mycoplasma species was used to target the conserved region of 16S rDNA intragenic spacer regions including those representing 90–95% of mycoplasma cell culture contaminations. This allows for the detection of a wide variety of mycoplasma strains, including fastidious strains that are difficult to detect even by conventional growth-based methods. We used universal Mycoplasma primer: forward primer—GGCGAATGGGTG AGTAACACG; reverse primer—CGGATAACGC TTGCGACCTATG.

Mycoplasma test was performed on cells before and after antibiotic application, and no mycoplasma infection was confirmed.

### Follow-up procedure

The patients were involved in a 12-month follow-up process after cell injection. We assessed neurological changes by the AIS score, functional recovery by the spinal cord independence measure (SCIM-III), and subjective changes along with adverse events (AE), presented in Table 2. A medical team including doctors, a physical therapist, and an occupational therapist assessed the patients for subjective changes, the severity, and the relevance of adverse events (AEs). All patients were monitored for adverse effects based on the Medical Dictionary for Regulatory Activities (MedDRA v. 18.1). The assessment of the changes in neuropathic pain and spasticity among the patients was based on subjective reports through exact history taking.

**Table 2:** Adverse events of the patients

Patient number		Adverse event						
		Fever	Numbness or tingling sensation	Facial flushing	Headache	General ache	Neuropathic pain	Spasticity
1	Before	−	−	−	−	−	−	−
	After 6 m	−	+	−	−	−	+	+
	After 12 m	−	+	−	−	−	−	↑
2	Before	−	−	−	−	−	−	−
	After 6 m	−	−	−	−	+	+	+
	After 12 m	−	−	−	−	+	+	↑
3	Before	−	+	−	−	−	−	−
	After 6 m	−	↑	+	−	−	−	+
	After 12 m	−	↑	+	−	−	−	↑
4	Before	−	+	−	−	−	−	+
	After 6 m	−	+	−	−	−	−	+
	After 12 m	−	+	−	−	−	−	+
5	Before	−	−	−	−	−	+	−
	After 6 m	−	−	−	−	−	+	−
	After 12 m	−	−	−	−	−	↓	−
6	Before	−	−	−	−	−	−	−
	After 6 m	−	−	−	−	−	−	−
	After 12 m	−	−	−	−	−	−	−
7	Before	−	−	+	−	−	+	+
	After 6 m	−	−	+	−	−	+	↑
	After 12 m	−	−	+	−	−	+	↑
8	Before	−	−	+	−	−	−	+
	After 6 m	−	+	+	−	−	−	↑
	After 12 m	−	+	+	−	−	−	↑
9	Before	−	−	−	−	−	−	+
	After 6 m	−	−	−	−	−	−	+
	After 12 m	−	−	−	−	−	−	+
10	Before	−	+	−	−	−	−	−
	After 6 m	−	↑	−	−	−	−	−
11	Before	−	+	−	−	−	−	+
	After 6 m	−	+	−	−	−	−	+
	After 12 m	−	+	−	−	−	−	+

+, presence of sign; −, absence of sign; ↑, increase in severity; ↓, decrease in severity

Furthermore, electromyography (EMG), nerve conduction velocity (NCV), magnetic resonance imaging (MRI), and urodynamic study (UDS) were conducted for all the patients at the baseline, 6 months, and 1 year after the intervention. We performed EMG-NCV based on the previous trials [8, 20] and to differentiate voluntary muscle contraction from reflex or involuntary spontaneous limb movement.

We also ensured that all the participants received standard therapy for SCI injuries such as regular rehabilitation programs.

### Statistical analysis

To study the significance of the changes in the clinical scales, the Wilcoxon rank test was used in SPSS 16.0 (IBM Crop., Armonk, USA). In all cases, the significance limit was placed on *p* < 0.05.

## Result

### Cell assessments

The extracted cells had the same characteristics as the cells we used in our previous study [15]. Cells isolated from the sural nerve were positive for S-100 marker, which indicated that these cells had the properties of SCs (Fig. 1A). MSCs were positive for CD73 and CD 105 and negative for CD45 and CD34 in flow cytometry analysis (Fig. 1B). In addition, the isolated cells could differentiate into adipogenic and osteogenic cells (data not shown).

**Fig. 1:** Results of bone marrow MSC and SC laboratory assessments. **A** S-100 immunocytological staining negative control. **B** S-100 immunocytological staining test. **C** The cell surface marker (CD73, CD105, CD45, and CD34) analysis through flow cytometry

### Adverse events

We observed some mild adverse events that based on medical team assessment; 38.46% were unlikely, 23.08% were possible, and 38.46% were probable AE. According to the MedDRA, the severity for each AE was mild. An increase in spasticity, numbness, or tingling sensation, and neuropathic pain was reported by 5, 4, and 2 out of 11 patients, respectively. Headache and facial flushing appeared in two patients after transplantation that was resolved spontaneously. Furthermore, none of the patients reported fever after injection (Table 2).

Other systemic complications such as anaphylactic shock, hypersensitivities, rush, or inflammation were not observed. Infectious complications associated with transplantation-like meningitis were not evident in the study. Since all AEs were mild, there was no need for medical treatment. However, the dose of the drug was increased for patients who already had a medical problem such as spasticity and had a mild increase after cell injection.

Although previous spinal instrumentation caused some worst effects on the visibility of images in the patients, MRI indicated no neoplastic overgrowth, syringomyelia, or pseudo-meningocele after transplantation (Fig. 2).

**Fig. 2:** Pre- and post-injection MRIs of patients with numbers 1, 6, and 8. **A** Patient number 1, pre-injection. **B** Patient number 1, 6-month post-injection. **C** Patient number 6, pre-injection. **D** Patient number 6, 6-month post-injection. **E** Patient number 8, pre-injection. **F** Patient number 8, 6-month post-injection

### AIS score evaluation

Sensory and/or motor improvement was evident in 9 patients according to the AIS assessment (in both score and motor and/or sensory level). Six patients experienced positive sensory changes in their AIS score (five patients also had changes in sensory level) and four patients had motor recovery (Table 1, Fig. 3). In our assessment, the cervical SCI patients showed more improvement rate in motor aspects (75% of the cervical and 14% of the lumbar-thoracic patients had motor improvement) and lumbar-thoracic SCI patients experienced more improvement rate in sensory AIS score (63% of the lumbar-thoracic and 50% of the cervical patients had sensory improvement) (Fig. 3). Among our patients, none of them showed AIS grade alteration from A to other grades.

**Fig. 3:** **A**–**C** Motor, sensory light touch, and pin-prick AIS scores in total population. **D**–**F** Motor, sensory light touch, and pin-prick AIS scores in cervical patients (*p-value ≤ 0.05)

In terms of the intensity of the changes, light touch AIS score alterations were approximately the same as the pinprick changes (11.6 ± 13.1 and 12 ± 13, respectively), and both were more than the motor score alterations (9.5 ± 3.3). Light touch scores among all the patients improved statistically significant after 6 and 12 months in comparison with pre-transplantation scores (*p*-value = 0.042 and 0.027, respectively). Score differences between the 6th and the12th months were not significant (*p*-value = 0.317). For pinprick, the results were the same as the light touch changes (*p*-value = 0.041, 0.027, and 0.317, respectively). The difference between the motor score in the pre-transplantation evaluation and 6- and 12-month follow-up was not significant (*p*-value = 0.068 and 0.066, respectively) (Fig. 3, Table 3).

**Table 3:** ASIA and SCIM III scores at different time points

Score subject		Population	Time	Mean	SD	***p***-value
ASIA	Motor score	Total study population	Before injection	37.54	17.58	–
			After 6 months	40.45	14.80	0.068
			After 12 months	41.00	14.58	0.066
		Thoracic patients	Before injection	50.00	00.00	–
			After 6 months	51.00	2.64	0.317
			After 12 months	51.28	3.40	0.317
		Cervical patients	Before injection	15.75	5.90	–
			After 6 months	22.00	1.63	0.109
			After 12 months	23.00	2.58	0.109
	Light touch	Total study population	Before injection	47.63	24.37	–
			After 6 months	50.54	24.46	0.042*
			After 12 months	51.80	25.74	0.027*
		Thoracic patients	Before injection	60.57	19.51	–
			After 6 months	63.71	17.12	0.109
			After 12 months	68.00	16.44	0.068
		Cervical patients	Before injection	25.00	12.05	–
			After 6 months	27.50	15.00	0.180
			After 12 months	27.50	15.00	0.180
	Pin prick	Total study population	Before injection	48.54	25.66	–
			After 6 months	51.63	25.71	0.041*
			After 12 months	53.00	27.00	0.027*
		Thoracic patients	Before injection	62.00	20.81	–
			After 6 months	65.42	19.13	0.102
			After 12 months	70.00	17.15	0.066
		Cervical patients	Before injection	25.00	12.09	–
			After 6 months	27.50	15.86	0.180
			After 12 months	27.50	15.86	0.180
SCIM III	Total score	Total study population	Before injection	28.9	12.99	–
			After 6 months	37.54	18.40	0.012*
			After 12 months	43.10	25.77	0.018*
		Thoracic patients	Before injection	37.14	6.28	–
			After 6 months	49.28	7.08	0.018*
			After 12 months	60.50	14.18	0.028*
		Cervical patients	Before injection	14.50	7.00	–
			After 6 months	17.00	12.00	0.317
			After 12 months	17.00	12. 00	0.317
	Self-care	Total study population	Before injection	8.00	5.53	–
			After 6 months	10.36	6.74	0.043*
			After 12 months	11.40	7.93	0.005**
		Thoracic patients	Before injection	11.71	2.49	–
			After 6 months	14.71	2.98	0.068
			After 12 months	17.16	2.48	0.042*
		Cervical patients	Before injection	1.50	1.00	–
			After 6 months	2.75	3.50	0.317
			After 12 months	2.75	3.50	0.317
	Respiration and sphincter management	Total study population	Before injection	17.18	5.89	–
			After 6 months	21.72	8.22	0.016*
			After 12 months	26.20	13.63	0.027*
		Thoracic patients	Before injection	19.57	4.64	–
			After 6 months	26.00	4.24	0.026*
			After 12 months	34.16	10.04	0.043*
		Cervical patients	Before injection	13.00	6.00	–
			After 6 months	14.25	8.50	0.317
			After 12 months	14.25	8.50	0.317
	Mobility	Total study population	Before injection	3.72	3.58	–
			After 6 months	5.45	4.78	0.039*
			After 12 months	8.90	12.81	0.043*
		Thoracic patients	Before injection	5.85	2.60	–
			After 6 months	8.57	2.63	0.039*
			After 12 months	14.83	13.77	0.043*
		Cervical patients	Before injection	0.00	0.00	–
			After 6 months	0.00	0.00	1.00
			After 12 months	0.00	0.00	1.00

Bold values indicate statistical significance (*p-value ≤ 0.05; **p-value ≤ 0.01)

### SCIM III changes

Regarding our SCIM III assessment, 8 out of 11 patients had some degrees of functional recovery, most of which were thoracic SCI patients. So, all the thoracic SCI patients experienced a positive change in SCIM III evaluation. Among the cervical SCI patients, only one patient (number 8) had improvement in the “sphincter management-bladder” item. The mean ± SD of the SCIM III changes was 21.2 ± 13.3, and among the SCIM III sub-scores, “respiration and sphincter management” (15 ± 9.9), “mobility” (9.5 ± 13.3), and “self-care” (6 ± 1.4) comprised the most of the score changes (Fig. 4).

**Fig. 4:** **A**–**D** Total, self-care, respiration and sphincter management, and mobility SCIM III scores in total population. **E**–**H** Total, self-care, respiration and sphincter management, and mobility SCIM III scores in thoracic patients (*p-value ≤ 0.05; **p-value ≤ 0.01)

Statistical analysis revealed that the patients experienced statistically significant progressive changes after every 6 months in SCIM III total score and its sub-scales (Fig. 4). Differences between the pre- and post-transplantation groups and between each post-transplantation group (cervical and thoracolumbar) were statistically significant in total SCIM III score, respiration and sphincter management, mobility, and self-care (*p*-values of changes after 6 months were 0.012, 0.043, 0.016, and 0.039, and *p*-values of changes after 12 months were 0.018, 0.005, 0.027, and 0.043, respectively). In thoracolumbar patients, our statistical evaluation revealed that the differences between pre-transplantation and 6 and 12 months were statistically significant (except self-care changes after 6 months, which were not significant). The *p*-values for changes of SCIM III score in thoracolumbar SCI patients after 6 and 12 months were 0.018 and 0.028, respectively (Table 3).

### Subjective outcomes

Our findings supported that the most remarkable positive, subjective improvement was in the trunk movement (in 8 patients) and equilibrium in standing/sitting positions (in 7 patients). Furthermore, three patients (patients with numbers 1, 3, and 5) experienced a reduction in the severity of constipation. We also observed that the two of our patients (numbers 1 and 9) claimed that they obtained the sensation of the filling bladder and rectum in the 6th and 12th months of their follow-up (patient number 1 acquired a sense of rectal filling in 12th months of follow-up). Furthermore, one patient had successful changes as the empowerment of voiding (patient number 5) (Table 4).

**Table 4:** Subjective changes of the patients

Patient number			Subjective changes								
		Trunk movement, 8	Equilibrium in sitting position, 7	Equilibrium in standing position, 7	Constipation	Urination sensation	Voiding	Consistency	Feeling of defecation	Bowel sphincter management	Regularity of bowel movement
1	Before	−	−	+	+	−	−	−	−	−	−
	After 6 m	−	−	↓	↓	+	−	−	−	−	+
	After 12 m	+	−	↓	↓	+	−	−	+	−	−
2	Before	+	+	+	+	−	−	+	−	−	+
	After 6 m	↑	↑	+	+	−	−	+	−	−	+
	After 12 m	↑	↑	+	+	−	−	+	−	−	+
3	Before	+	+	+	+	−	−	−	−	−	−
	After 6 m	↑	↑	↓	↓	−	−	−	−	−	−
	After 12 m	↑	↑	↓	↓	−	−	−	−	−	−
4	Before	−	−	−	−	−	−	−	−	−	−
	After 6 m	−	−	−	−	−	−	−	−	−	−
	After 12 m	−	−	−	−	−	−	−	−	−	−
5	Before	+	+	+	+	−	−	−	+	+	−
	After 6 m	↑	+	+	+	−	+	−	+	+	−
	After 12 m	↑	+	↓	↓	−	+	−	+	+	−
6	Before	+	−	−	−	−	−	−	−	−	+
	After 6 m	↑	+	−	−	−	−	−	−	−	+
	After 12 m	↑	↑	−	−	−	−	−	−	−	+
7	Before	+	−	−	−	−	−	−	−	−	−
	After 6 m	↑	+	−	−	−	−	−	−	−	−
	After 12 m	↑	↑	−	−	−	−	−	−	−	−
8	Before	+	−	+	+	−	−	−	−	−	−
	After 6 m	↑	+	+	+	−	−	−	−	−	−
	After 12 m	↑	↑	+	+	−	−	−	−	−	−
9	Before	−	−	−	−	−	−	−	−	−	−
	After 6 m	+	+	−	−	+	−	−	+	−	−
	After 12 m	↑	↑	−	−	+	−	−	+	−	−
10	Before	+	−	+	+	−	−	−	−	−	+
	After 6 m	+	+	+	+	−	−	−	−	−	+
11	Before	−	−	−	−	−	−	−	−	−	−
	After 6 m	−	−	−	−	−	−	−	−	−	−
	After 12 m	−	−	−	−	−	−	−	−	−	−

+, presence of sign; −, absence of sign; ↑, increase in severity; ↓, decrease in severity

UDS assessment of patient number 5 also supported this change. Pre-transplantation UDS of the patient revealed the presence of uninhibited contraction (no voiding), maximum detrusor pressure of 55cmH_2_O, maximum flow during cytometry less than 1 cc/s, and post-voiding residue of 314 cc. Post-transplantation UDS changed to maximum detrusor pressure of 15 cmH_2_O, maximum flow during cytometry of 3.3 cc/s, a post-voiding residue of 410 cc, and voided volume of 40 cc.

## Discussion

The present study showed that autologous SC and bone marrow-derived MSC transplantation at the subacute stage of SCI could reveal statistically significant improvement in sensory and neurological function among the patients. Describing changes of patients with spinal cord injury includes many aspects consist of neurological, functional, and quality of life changes. The distinction of these improvements could be presented by AIS and SCIM III scores which indicated neurological and functional changes, respectively. Also, there is a difference between statistically significant and clinically significant. Although some changes in the AIS score are statistically significant, the transplantation did not change the AIS grade, and therefore, no clinically significant improvement could be considered. Furthermore, the changes in SCIM score which is statistically significant could be considered clinically significant because SCIM is a functional scale. In the present study, 75% of the cervical patients showed some degrees of motor improvements and 50% of them had sensory changes. But, thoracolumbar SCI patients experienced more improvement rate in sensory AIS score (63% of the patients) and less in the motor score (14%). Two patients obtained the sensation of the bladder and rectal filling and one patient claimed that he acquired the ability of voluntary voiding. There were no systemic nor serious complications such as fever, anaphylactic shock, hypersensitivities, rush, or inflammation after autologous transplantation. Also, radiological images showed no neoplastic overgrowth, syringomyelia, or psuedomeningocele, which documents the safety of using this cell combination therapy at the subacute stage.

The current clinical trial used the combination of autologous SC and bone marrow-derived MSC transplantation because of the multi-faceted inhibitory nature of the CNS lesion [22]. After spinal cord injury, multiple changes occur in damaged tissues that require various treatment strategies like neuroprotection, axonal regeneration promotion, and rehabilitation [23].

Since one of the issues following spinal cord injury is an inflammatory environment, previous treatment strategies have focused on reducing inflammatory responses. In the past, only high-dose methylprednisolone has been shown as the standard of care and has limited effectiveness for regenerating the spinal cord [24].

Cell transplantation is a targeted new promising therapeutic strategy for spinal cord regeneration based on a series of animal and clinical studies, and it has been previously reported that stem cells have a potential effect on the SCI treatment [20, 25, 26]. The safety and clinical application of SCs and MSCs separately have been reported in the treatment of SCI patients [7, 8, 27, 28]. MSCs are an appropriate source for cell therapy due to their ability of high growth rate, low immunogenicity, and favorable ethical profile [29]. Also, MSCs could enhance and support neurite outgrowth, axonal survival, and remyelination [30]. In spite of the beneficial effects of MSC transplantation, according to the previous findings, their remyelinating ability is inadequate in SCI patients [15]. So far, some studies have performed combination therapies for spinal cord regeneration; using two types of effective cells (SCs and MSCs) for spinal cord regeneration is one of these combination methods [23, 31, 32]. In our previous work, we reported the safety of SCs and MSCs combination therapy in the damaged chronic human spinal cord with no new deficit or adverse effect in the patients during short- and longer-term assessments [15]. Park et al. evaluated the therapeutic effects of autologous bone marrow cell transplantation in conjunction with administering granulocyte macrophage-colony stimulating factor (GM-CSF) in six complete SCI patients and reported neurologic improvements in AIS grades (from A to C) in five patients [33].

The delivery time of the stem cells after spinal cord injury is important for a better prognosis. This is because oligodendrocyte death and myelin loss after SCI are not a static phenomenon and demyelination continues and increases up to at least 450 days post-injury [33]. Generally, 12–18 months post-injury optimally correspond with the natural history of neuro recovery; this time is the golden time for supporting and improving neuro recovery and promoting conditions for the long-term maintenance of health and function [19]. In spite of promising results in chronic SCI patients after cell therapy [13, 34, 35], it seems that the sub-acute phase of stem cell transplantation after SCI may lead to better results [34]. The study by Yoon et al. reported improvement in AIS grade of 30.4% of the acute and subacute treated patients (AIS A to B or C), whereas no statistically significant changes were observed in the chronic patients. The majority of their study population had cervical injuries; nevertheless, they did not report the changes separately regarding the cervical and thoracic SCI patients [8]. Some differences between our results and theirs could be explained by the different composition levels of injury and cell combination therapy in our study [35].

Among the 11 patients, one reported improvement in urination management after cell therapy. Likely, Jiang et al.’s study [12] showed 80% of patients experienced recovery of urinary function. Nevertheless, Kishk et al. reported that no one in the treated or control groups reached the complete recovery of bladder control [20]. This controversy in the results could arise from different evaluation systems in each study. Despite the importance of urinary problems in SCI, there was a lack of comprehensive study for assessing cell transplantation in human subjects.

Neuropathic pain is one of the irritable complications that increases after cell transplantation, so is observed in some patients based on our study and other previous works [20, 36]. One of the possible reasons for neuropathic pain after cell therapy may be due to MSC differentiation into astrocytes which could lead to increased CGRP-positive sprouting and a consequent hypersensitive state [21, 37]. Because of the small sample size and lack of a control group, we could not conclude that the intrathecal injection of this combination cell therapy may increase neuropathic pain. So, clinical trials with larger volume sizes and control groups are needed for definitive comment on this topic.

In the present study, we used SC and MSC combination therapy in complete subacute SCI subjects to assess the safety and possible outcomes of this intervention. Unlike our previous findings [13], the results of this treatment in subacute patients were promising for the patients’ rehabilitation. Our data were in reasonably close agreement with the hopeful effects of combination cell therapy in sensory, motor, and functional status of subacute SCI patients alongside the positive subjective changes like empowerment in trunk movement, equilibrium in standing/sitting position, and sensation of the bladder and rectal filling. According to our limitations, we suggest a clinical trial with a large number of patients to unveil the effects of this kind of therapy on the suitable subgroups of SCI patients.

The nature of neural regeneration of SCI encountering many factors which mostly presents in the golden time for neurological improvements over the first 1–2 years post-injury. This fact is one of the important parameters affecting our results and limits our conclusion.

## Conclusion

It seems that the combination of autologous SC and bone marrow-derived MSC transplantation at the subacute stage of SCI could significantly improve sensory and neurological function among the patients. Also, there were no systemic nor serious complications after autologous transplantation. This study is a phase 1/2 trial that aimed to provide the important information needed for the design of each respective trial phase. It is a preliminary study on the safety and feasibility of stem cells on spinal cord injury and to develop a preliminary sense of potential efficacy that its results can be used as a guide for configuring future studies because clinical efficacy could not be made without a randomized controlled clinical trial.

## Data Availability

Researchers could submit their research proposals to the corresponding author to access datasets of this clinical trial.

## Abbreviations

SCI: Spinal cord injury
MSCs: Mesenchymal stem cells
SCs: Schwann cells
ASIA: American Spinal Injury Association Impairment Scale
SCIM: Spinal cord independence measure
AE: Adverse event
EMG: Electromyography
NCV: Nerve conduction velocity
MRI: Magnetic resonance imaging
UDS: Urodynamic study
GBD: Global burden of diseases
GMP: Good Manufacturing Practice
FBS: Fetal bovine serum
CSF: Cerebrospinal fluid
PCR: Polymerase chain reaction
CNS: Central nervous system
GM-CSF: Granulocyte macrophage-colony stimulating factor
DMEM/F12: Dulbecco’s modified Eagle medium/Nutrient Mixture F-12
